The article "The Biomechanical Relationship between Hallux Valgus Deformity and Metatarsal Pain" was published in 2020. Journal: J Healthc Eng.

# The Biomechanical Relationship between Hallux Valgus Deformity and Metatarsal Pain

**DOI:** 10.1155/2020/8929153

**Published:** 2020-03-25

**Authors:** Cheng Chang, Qing-Fu Wang, Jun-Chao Guo, Duo-Duo Li, Yu-Bo Fan, Jian-Min Wen

**Affiliations:** ^1^Beijing University of Chinese Medicine, Beijing, China; ^2^Wangjing Hospital, China Academy of Chinese Medical Sciences, Beijing, China; ^3^Beijing Key Laboratory of Rehabilitation Technical Aids for Old-Age Disability, Key Laboratory of Human Motion Analysis and Rehabilitation Technology of the Ministry of Civil Affairs, National Research Center for Rehabilitation Technical Aids, Beijing, China; ^4^Key Laboratory for Biomechanics and Mechanobiology of Ministry of Education, Beijing Advanced Innovation Centre for Biomedical Engineering, Beihang University, Beijing, China

## Abstract

Metatarsal pain is a common pathological outcome in patients with a hallux valgus (HV) deformity. However, the relationship between the degree of HV deformity and metatarsal pain has not been systematically examined. The purpose of the present study was to investigate the correlation between metatarsal pain and the degree of HV deformity. Between October 2017 and September 2018, 512 HV patients (944 feet) participated in an evaluation of their HV angle (HVA) using X-ray images. The participants were divided into four groups corresponding to their HVA (<15°, 15° to 20°, 21° to 40°, or >40°). Load rate, impulse, contact duration, and contact area were measured and recorded as dynamic gait parameters using the RsScan system. Data were evaluated using SPSS statistical software. The visual analog scale (VAS) was used to assess metatarsal pain. For the four HV deformity groups, the peak value of impulse and contact duration was concentrated on the second and third metatarsals (Meta2 and Meta3) (*P* < 0.05); contact area was also shown on metatarsals 1, 2, and 5 (*P* < 0.05). Metatarsal pain on Meta2 had the highest VAS score (VAS: 6.57), followed by Meta3 (Mean VAS: 5.72). In the HV > 40° group, the load location on Meta2 was transferred to Meta1. The percent of pain attributed to Meta2 and Meta3 was also increased in this group. These findings illustrated that metatarsal pain was primarily located on Meta2 and Meta3 in the different degrees of HV deformity. This information can provide the location to target for pain relief and help guide further rehabilitation.

## 1. Introduction

Hallux valgus (HV) is a common condition in females and consists of complex malposition of the first metatarsal (Meta) and lateral deviation of the great toe [1]. The prevalence rate of 12–33% is much high because of constrictive or high heel shoes popular among women [2]. Compression of the skin and subcutaneous tissues between the footwear and foot exacerbates the bunion [2] and forms a protrusion tuberosity on the medial first metatarsal head [3]. As a result, this condition seriously affects the gait and foot health of HV patient [3].

Forefoot pain in HV patients has been reported by previous studies [4, 5]. Contacting the ground with the forefoot for a long period of time will induce medial pain in the first metatarsophalangeal joint [4]. The main reason for this pain is that the medial ligamentous tension is weakened in early HV patients. With increasing severity in the degree of HV deformity, the phalanx slowly drifts into a valgus position and the metatarsal head escapes from the sesamoid platform [6]. The medial articular cartilage on the first metatarsal head thus loses the normal contact relation with the proximal phalanx and is no longer subjected to the normal pressure [6, 7]. Toe spacer pads [8], rehabilitation training [9], and orthotic footwear [10] all have been shown to improve the pressure to relieve pain from the first metatarsal. However, physical therapy has also shown insufficient pain relief [5]. This may be due to inaccurate loading location between the first ray and footwear [2]. Previous studies have also demonstrated the effect of the plantar callosities on metatarsal regions with aggravated HV [4, 6, 7].

Many studies have suggested that plantar pressure is the main cause of metatarsal pain in HV patients [10–14]. Hutton and Dhanendran found that the third metatarsal had the higher peak pressure in an investigation of HV pain [11]. Marta et al. found that the Meta2 region had the highest pressure in forefoot regions [12]. It was reported that the force loading on Meta1–3 was higher than on Meta4–5 [13]. Francesc et al. measured visual analog scale (VAS) scores in different metatarsal pain regions. It was found that the main pain regions were on Meta2–3 [14]. Other research has found that increasing severity of HV degree results in increased load on the metatarsal heads [12]. This may be a result of the compression of the skin between footwear and the bunion protrusion [2], the abnormal contact relation of the articular cartilage [7], or extensor hallucis longus tendon dysfunction [6]. However, the relationship between metatarsal pain and the degree of HV severity has not been systematically examined.

Therefore, the aim of this study was to investigate the relationship between the degree of HV severity and metatarsal pain using biomechanical testing, medical images, and software.

## 2. Methods

### 2.1. Sample

The 512 patients with HV (944 feet) from Rehabilitation Hospital, National Research Center for Rehabilitation Technical Aids, participated in this study between October 2017 and September 2018. Informed consent was obtained from each participant, and the experimental procedures were approved by the ethical committee of hospital. The VAS score for Meta regions' pain was administered and recorded by a professional physician [15]. HV angle (HVA) of 944 feet during full weight-bearing was recorded using X-ray images and measured using MIMICS10.01 software (Materialise, Belgium). The participants walked barefoot on the pressure plate at an adaptive speed. The plate was 2 m by 0.4 m in dimension with a sampling frequency of 250 Hz. The corresponding plantar partitions were divided into 10 regions (Toe1, Toe2–5, Meta1, Meta2, Meta3, Meta4, Meta5, Forefoot, Midfoot, and Hindfoot), and pressures were also recorded during a gait cycle using the RsScan system (RsScan, Belgium) [16]. A minimum of three valid trials per participant were recorded and collected [17].

The 944 feet were further divided into four groups according to HVA severity. Four levels of HV (the levels of HV are defined by the hallux valgus angle) were classified into mild, mild-moderate, moderate, and severe [18]: group 1 with mild (HVA ≤ 15°), group 2 with mild-moderate (15° < HVA ≤ 20°), group 3 with moderate (20° < HVA < 40°), and group 4 with severe (HVA ≥ 40°) [18, 19] (Figure 1). The percentage of female patients was 87.0%, 96.0%, 95.9%, and 94% in group 1 to group 4, respectively. The gender distribution of HV patients was consistent with previous research [20] (Table 1).

### 2.2. Data Analysis

Region of the forefoot was divided into 5 anatomical regions using the RsScan software system. All division results were appropriately adjusted by the software system. Each parameter was calculated using the dense sensor array in the RsScan system, instead of using a calculation based on a single-sensor grid within a region. Two hundred data points from the pressure plate were recorded using the dense sensor array. Test data were interpolated using piecewise cubic spline interpolation. The total force (*F*_*A*_) was calculated using the total number of data frames (before interpolation) during a single trial. The frame number was proportionate to the foot contact duration, the percentage of which is relatively constant in a gait cycle over various walking speeds. The data were normalized by the *F*_*A*_ divided by the total number of data frames. This test method is superior to the calculation of a single-sensor grid within a region [17].

We further derived various parameters for HV assessment. Load rate represented the loading conditions of the metatarsal regions in a short contact time. This relative measure was defined as *F*_Meta1–5_/*F*_*A*_ and was relevant to HV patients as an important feature of Meta1–5 loading and as a reference of HV patient pain during foot contact. The loading condition was selected because it had higher reliability than peak pressure. The impulse of loading could be characterized equally well with either force or pressure [17].

An independent one-sample *T*-test was used to analyze the differences between four groups with a significance level at 0.05. The parameters of the load rate, impulses, contact area, and pain index were focused on a comparison of the Meta1–5 regions during contact ground and lift-off of the forefoot. In addition, the percent of pain was calculated as each metatarsal's pain score divided by the total pain score in each group of patients.

## 3. Results

Figure 2 shows the peak value and location of load rate in Meta1–5 for the four groups. The load location was concentrated on the Meta2 region in groups 1–3 but was shifted to the Meta1 region in group 4. The load locations of the first, second, and third peak values were all on Meta1–3 in all four groups, with no significant differences between groups (*P* < 0.05).

The impulse (Figure 3(a)), contact duration (Figure 3(b)), and contact area (Figure 3(c)) of Meta1–5 in the four groups are presented in Figure 3. For the peak and second peak value locations of Meta2–3, there were no differences in the four groups. However, the third peak value location was concentrated on Meta4 in group 1–3 and was shifted toward Meta1 in group 4. With increasing degree of HV severity, the impulse of Meta1–5 had a significant upward trend (*P* < 0.05) (Figure 3(a)). For the different HV pain patients, the contact duration of Meta2 and Meta3 were not different (Figure 3(b)) (*P* < 0.05). For the contact area of the Meta1–5 regions, the order of peak value location was the first, second, and fifth metatarsal regions in all four groups (Figure 3(c)) (*P* < 0.05).

The percent of pain in the Meta1–5 regions for the four groups is presented in Figure 4. Meta2 was the region where patients from all groups had highest proportion of pain, followed by the Meta3 (Table 2). The percentage of pain in Meta2 and Meta3 was similar across all four groups (*P* < 0.05). The proportion of patients with pain in Meta2 and Meta3 was 50.63% and 68.7% of total feet, respectively. The mean VAS scores of Meta2 and Meta3 pain were 6.57 and 5.72 (Table 2). In addition, the pain locations of Meta2 and Meta3 showed an upward trend with increases in HV severity degree (Figure 4).

## 4. Discussion

In this study, 512 HV patients participated in a biomechanical investigation between the degree of HV severity and metatarsal pain. In clinical practice, HVA as a parameter could directly reflect the pathological behavior of the first ray [18, 21]. The degree of deformity of HV has typically been assessed by previous studies using the angle of the first ray [5, 9, 18, 21, 22]. In this study, X-ray images and plantar pressure measurement were used to investigate HV deformity. These methods had been widely used in previous research of HV patients [21, 22]. Our results showed that females had a higher incidence rate of HV, and the percentage of female patients was 87.0%, 96.0%, 95.9%, and 94% from group 1 to group 4, respectively. There was no significant different in this rate between groups, which is consistent with the gender distribution of HV patients in the literature [6, 20, 21] (Table 1).

In clinical practice, plantar pressure has typically been used to assess foot function of HV patients during gait and other activities [23]. The static and dynamic plantar pressures directly show the tendencies in different plantar loading condition [23]. One study found that higher peak forces were concentrated on the third metatarsal region and the great and second toes [11]. The forces on Meta1–3 have also been shown to be higher than Meta4 and Meta5 [13]. Nevertheless, Martinez-Nova et al. reported that the highest pressures were on the Meta2 head [12]. This is consistent with the peak load rate location being on Meta2 in the present study (Figure 2). One possible reason is that the extensor hallucis longus tendon followed the deviation of the phalanx [6], and the alignment of the first ray was altered by the internal tissue tension [11, 12]. The flexor hallucis longus also acts as an adductor to disable function. Musculoskeletal disorders extrude the second metatarsal regions and aggravate HV deformity [12], which was also the main source of Meta2 pain in our study (Table 2).

With an increase in the degree of HV deformity (group 4), the load location was shifted from Meta2 toward Meta1 (Figure 2). It has been previously demonstrated that the load rate of Meta1 is improved in normal gait [12]. This pathological behavior was from an alteration of muscle vector imbalance that led to medial rotation or pronation of the hallux [11, 12]. This resulted in severe compression between the skin and subcutaneous tissues, which would lead to a sharp increase in Meta2 pain (Figure 4). This is also in accordance with the higher VAS scores of Meta2 (6.57) and Meta3 (5.72) (Table 2). However, the previous literature report showed that the VAS index of Meta was slightly more than 5 [24]. This is because the literature has primarily examined HV postoperation pain rather than investigation of preoperation pain. There was no difference in pain between the Meta2 and Meta3 regions in four groups (*P* < 0.05).

Corresponding to the higher pain percentage of Meta2–3 in the four groups (Figure 4), the VAS pain score increased significantly with increased severity of HV deformity (Table 2). Previous studies found a positive correlation between HV deformity and metatarsal pain levels [18, 24]. Increasing HV severity was also significantly associated with greater Meta pain and decreased foot function [25]. The higher percentage of pain at Meta2 and Meta3 (Figure 4) was in line with the higher VAS scores (Table 2).

Our results not only confirmed the positive correlation of the previous research [25] but also confirmed the location of metatarsal region pain. At the same time, the peak load rate of Meta2 (Figure 2) and the peak impulse and contact duration of Meta2 and Meta3 (Figures 3(a) and 3(b)) were not significantly different between the four groups. The previous studies had shown greater loading on Meta2 and Meta3 during normal gait of HV patients [21, 22, 26]. It was also shown that the contact time had the tendency of increase between Meta2–3 and the plantar foot in the gait of HV patients [25, 26]. Therefore, these results indicate that pain on Meta2 and Meta3 is nearly universal, regardless of HV patient severity. This provides information to determine whether operation or physical therapy would best benefit the further treatment of a patient with HV.

In addition, we also found that there were no significant differences in pain between Meta1 and Meta4–5, regardless of HV severity (Figure 4). Compared with the higher value of Meta2–3, the lower impulse (Figure 3(a)) and contact duration (Figure 3(b)) of Meta1, 4, and 5 suggested that the decreased loading of Meta4–5 had a same tendency in four groups [13]. Moreover, the greatest contact area of Meta1–5 was at the first, second, and fifth metatarsal regions across all groups, with no significant differences (Figure 3(c)). With increasing severity of HV, it has been indicated that the musculoskeletal disorder was subjected to tension of short flexors and muscle vectors imbalance [11, 12]. The contact area was not bound to phalanx valgus and metatarsal head escape [6]. In terms of contact area, it was effective to reduce metatarsal pain changing the touchdown area of the forefoot. Therefore, this would propose a suggestion for footwear design for HV patients.

As a statistical method for HV patients, there were some limitations in the present study. First, although the total sample was large, the percentage outcomes may have the negative effect because of the unequal subjects in four groups. Second, we did not consider the difference of the individual foot, such as the width of forefoot in transverse. Whether this factor was unreasonable for the metatarsal pain was debatable.

## 5. Conclusion

In this study, the biomechanical behaviors of HV based on a large sample were quantified and evaluated using X-ray images, a plantar pressure test system, and VAS score. We compared differences in gait parameters between four groups of varying HV deformity. We found that the longer contact duration of Meta2–3 had a higher load rate and impulse with increasing HV severity. Meta2 and Meta3 were the main regions of pain, regardless of HV severity. This information can provide the location to target for pain relief and help guide further rehabilitation.

## Figures and Tables

**Figure 1:** Diagram of four group patients: (a) mild HVA; (b) mild-moderate HVA; (c) moderate HVA; and (d) severity HVA.

**Figure 2:** Load rate of five metatarsal regions in four different groups.

**Figure 3:** Five metatarsal regions in four groups (a) Impulse (It represents that the process of mutation is from the metatarsal contact ground to return its original state); (b) contact duration; and (c) contact area.

**Figure 4:** Percent of Meta1–5 regions' pain in HV patients of four groups.

**Table 1:** The data description of the four groups' participants (mean within each group were shown).

Characteristics	Group 1	Group 2	Group 3	Group 4
Number of feet HVA	*N* = 77 ≤15°	*N* = 101 15°∼20°	*N* = 617 20°∼40°	*N* = 149 >40°
Sex (male/female)	10/67	4/97	25/592	9/140
Age (years)	52.12 ± 14.35	48.65 ± 13.02	51.54 ± 13.64	55.42 ± 14.17

**Table 2:** Number and VAS score of Meta1–5 in HV patients of four groups.

Groups	Meta1	Meta2	Meta3	Meta4	Meta5
	Feet (%)	Feet (%)	Feet (%)	Feet (%)	Feet (%)
Group 1 (*N* = 77)	0 (0%)	8 (10.4%)	2 (2.6%)	0 (0%)	2 (2.6%)
Group 2 (*N* = 101)	1 (1%)	45 (44.6%)	17 (16.8%)	1 (1%)	5 (5%)
Group 3 (*N* = 617)	27 (4.4%)	335 (54.3%)	101 (16.4%)	23 (3.7%)	16 (2.6%)
Group 4 (*N* = 149)	10 (6.7%)	90 (60.4%)	51 (34.2%)	12 (8.1%)	5 (3.4%)
Mean VAS score	3.42	6.57	5.72	2.64	1.38
*P* value	0.026	0.0007	0.0008	0.071	0.254

## Data Availability

In our manuscripts, we declare that the data sharing would allow other researchers to verify the results of an article.
